The article "The Accessibility of Educational Public Service Facilities with Two-Step Mobile Search Taking Hetao District of Ganzhou City as an Example" was retracted in 2023. Reasons: unreliable results or conclusions; concerns about the data; concerns about the peer review; concerns about the citations.

# The Accessibility of Educational Public Service Facilities with Two-Step Mobile Search Taking Hetao District of Ganzhou City as an Example

**DOI:** 10.1155/2022/5646260

**Published:** 2022-08-11

**Authors:** Xibin You, Yuanfang Fu, Tingting Liu

**Affiliations:** ^1^Nanling Revitalization and Development Institute, Shaoguan University, Shaoguan 521005, Guangdong, China; ^2^Key Laboratory of Poyang Lake Wetland and Watershed Research Ministry of Education, Jiangxi Normal University, Nanchang 3300027, Jiangxi, China; ^3^Art and Design Institute, Shaoguan University, Shaoguan 521005, Guangdong, China

## Abstract

By using the two-step mobile search method of time and distance cost combined with Internet map data, taking the old urban district of Ganzhou city as research object, the spatial accessibility of primary and secondary schools from residential sites to residential areas was studied. The research shows that the reachability of primary and secondary schools in the old urban district of Ganzhou city is low, and most of the population fails to enjoy better education resources and the spatial distribution of education resources is not balanced. The reachability of primary education resources is high in geospatial area. The gathering area is the intersection of Ganjiang Street and Jiefang Street. The low-value areas are mainly the southwestern part of Nanwai Street and the northwestern area of Dongwai Street. The reachability of education resources shows a decreasing trend from the center to the surrounding areas. The education resources are concentrated in Ganjiang Street. Compared with traditional methods, the two-step mobile search method using Internet map data can more effectively and accurately reflect the accessibility of residential areas to primary and secondary schools in real time and can obtain the real conditions of traffic and roads more conveniently and also more accurat data acquisition.

## 1. Introduction

Nowadays, the social contradiction has been due to unbalanced and inadequate development. It affects social development and also hinders the rapid pace of realizing the Chinese dream. Education is the starting point of social justice and has always been widely emphasized in the community. However, the traditional space configuration method of educational facilities is seperated from what has gradually failed to meet the needs of social development and urban planning because of lack of touch with the needs of residents. In recent years, space configuration accessibility is widely used in the spatial configuration of educational facilities, where accessibility refers to the ease of one point to another, taking into account the distance, cost, and time between the supply point and the demand point [1]. Foreign scholars first introduced spatial accessibility to the field of public services and carried out a large number of empirical studies on urban public service facilities such as educational facilities, medical facilities, elderly facilities, parks, and green spaces. For example[2], Dai has studied the accessibility of public green spaces in the black residential areas of Detroit [3, 4]; Schuurman and McGrail conducted an accessibility analysis of primary medical service facilities [5, 6]. In China, Dadao introduced accessibility from abroad and analyzed public service facilities [7]. Wang et al. proposed a facility accessibility calculation method based on the GIS gravity model and calculated the service range of hospital service facilities of Pudong New Area in Shanghai [8]. Chen evaluated the accessibility of primary schools with distance attenuation and nondistance attenuation in Zhuhai district, Guangzhou [9]; Xiao used the spatial analysis function of GIS to assess the accessibility and fairness of secondary school education facilities in Xi'an and it was evaluated [10]. Liu used a two-step mobile search method to study the accessibility of medical and health-care facilities in Beijing [11]. Song introduced the research method of spatial accessibility through the use of the potential model and the two-step mobile search method in education and medical service facilities, respectively [12]. Che also summarized the methods of spatial accessibility, and analyzed their advantages and disadvantages [13]; Deng evaluated the accessibility and accessibility of medical facilities in Shizhu County, Chongqing with an improved two-step mobile search method [14].

The article "The Accessibility of Educational Public Service Facilities with Two-Step Mobile Search Taking Hetao District of Ganzhou City as an Example" was retracted in 2023. Reasons: unreliable results or conclusions; concerns about the data; concerns about the peer review; concerns about the citations.

At present, there are many methods to study the accessibility of public service facilities. Among them, the two-step mobile search method comprehensively considers the relationship between supply and demand and can more accurately reflect the distribution of spatial accessibility. In recent years, it has been widely used in the accessibility measurement of foreign primary medical care and continuously improved [6, 15, 16]. For example, Luo et al. [17]divided the travel time between supply and demand points into segments and assigned different weights. In fact, the most important improvement of this method in recent years is that the use of spatial scope changes due to changes in its actual population and services. McGrail et al. [18] proposed an improved two-step mobile search method to improve its accuracy in evaluating public service facilities. In China, Cheng [19], Hu [20], Tao [21, 22], Wei [23], and Zhang [24]used a two-step mobile search method to search for parks, green spaces, medical facilities, and elderly care facilities, The spatial accessibility of public service facilities such as tourist attractions is analyzed.

The article "The Accessibility of Educational Public Service Facilities with Two-Step Mobile Search Taking Hetao District of Ganzhou City as an Example" was retracted in 2023. Reasons: unreliable results or conclusions; concerns about the data; concerns about the peer review; concerns about the citations.

Now, of big data technology changes with each passing day, more and more data can be obtained from public online channels. It captures the point of interest data and route planning data provided by Baidu Map API as basic data with python programming language to study the connection between the community and the education service center by using walking and driving as the mode of travel. Compared with traditional data collection methods, Baidu Map API interface technology is more convenient and faster to obtain data and can collect a large amount of data at one time. By obtaining the required data such as the location of the community and its health service center, and the travel situation between the two points, the traffic accessibility of the educational service facilities in Ganzhou can be further explored with the two-step mobile search method.

## 2. Study Area

Ganzhou City is located in the south of Jiangxi Province at the junction of the four provinces of Jiangxi, Guangdong, Fujian, and Hunan (Figure 1). Ganzhou is a national historical and cultural city that is 2,000 years old. As an important Hakka gathering area, Ganzhou has a strong tradition of advocating culture and education. In the old district, there are seven secondary schools, such as No. 1, No. 2, No. 3, No. 4, No. 7, Affiliated Secondary School of Gannan Normal University, and Wenqing Experimental School in the old city and 15 primary schools include Cha'e Temple School, Zhongshan Road School, Xijin Road School, Dagonglu No. 1 School, Dagonglu No. 1 School (north district), Dagonglu No. 2 School, Houde Road Primary School, Wenqing Road Primary School, Binjiang No. 2 School, Binjiang No. 2 School, Binjiang No. 2 School (Jiaxuan Road Campus), Hongqi Avenue No. 2 School, Hongqi Avenue No. 2 Primary School (Huangwuping Road Campus), Tianzhushan Primary School, and Baiyun Primary School (Figure 2).

## 3. Data Sources and Research Methods

### 3.1. Data Sources

#### 3.1.1. Vector data

Vector data files in urban space research have a fundamental role. The vector data used in this article are all in shapefile format data. Due to the lack of existing vector data, the vector data in this article are obtained by artificial vectorization methods to ensure the timeliness and usability of the data.

#### 3.1.2. Internet Data

All travel data in this article comes from the route planning API in Baidu Maps API. Compared with traditional network analysis and buffering methods, it is convenient to obtain data based on the Internet map method without the road network land. At the same time, more accurate travel data for different modes of transportation can be obtained, and the obtained data are all real actual data, which takes into account real conditions such as traffic jams and has strong timeliness.

The article "The Accessibility of Educational Public Service Facilities with Two-Step Mobile Search Taking Hetao District of Ganzhou City as an Example" was retracted in 2023. Reasons: unreliable results or conclusions; concerns about the data; concerns about the peer review; concerns about the citations.

The data acquisition steps are as follows:

- Application key(ak)
- Set parameters through python programming language
- Receive the json data returned by Baidu map through the request spackage
- Data cleaning and storage

The related program code is shown in Figure 3.

### 3.2. Research Method

#### 3.2.1. Two-step Mobile Search

The two-step mobile search is an improved model of the mobile search, which overcomes the distance between the supply and demand in the space scope with the mobile search that may exceed the set distance or the facilities do not serve the demands of the region fully. The main idea is the first is to search for demand point *k* within the space scope of the supply point *j* by path-planning function of Baidu Map API to *j*, and calculate the supply-demand ratio *R*_j_ [15, 16].

(1) $$\begin{array}{c} R_{j}=\frac{s_{j}}{\sum_{j\in }\left(d_{ij}\leq d_{0}\right)D_{k}}. \end{array}$$

Here, *d*_ij_ is the distance or time between *k* and *j* measured by Baidu API, and *D*_*k*_ is the residents (*d*_ij_ ≤ *d*_0_) demand of the search area, and *S*_*j*_ is the total supply of point *j*.

The second is, in each demand point *i*, with path-planning function of the Baidu Map API, search for all supply points *j* within the scope of *i* space *d*_0_ and add up all the supply-demand ratios *R*_*j*_ to get the reachability *A*_*i*_^*F*^ of point *i*.

(2) $$\begin{array}{c} A_{i}^{F}=\sum_{j\in \left(d_{ij}\leq d_{0}\right)}Rj=\sum_{j\in \left(d_{ij}\leq d_{0}\right)}\left[\frac{s_{j}}{\sum_{j\in \left(d_{ij}\leq d_{0}\right)}D_{k}}\right]. \end{array}$$

Here, *d*_ij_ is the distance between *i* and *j*, and *R* is the supply-demand ratio of the supply point *j* in the *i* search area ( *d*_ij_ ≤ *d*_0_). AF is the accessibility of the residential area [24].

#### 3.2.2. Spatial Autocorrelation Index

The spatial autocorrelation index can be calculated by formula

(3) $$\begin{array}{c} I=\frac{n\sum_{i=1}^{n}\sum_{j=1}^{n}C_{ij}\left(x_{i}-\bar{x}\right)\left(x_{j}-\bar{x}\right)}{n\sum_{i=1}^{n}\sum_{j=1}^{n}C_{ij}{\left(x_{i}-\bar{x}\right)}^{2}}. \end{array}$$

Among them, *I* is the global spatial autocorrelation index. The greater the absolute value, the higher the similarity degree of the element and neighborhood element. N is the number of space units; *C*_*ij*_ is the relationship of space units between I and J. If the two sides are common adjacent, the value is 1; otherwise, the value is 0; $\bar{x}$is the mean of region attribute.

The article "The Accessibility of Educational Public Service Facilities with Two-Step Mobile Search Taking Hetao District of Ganzhou City as an Example" was retracted in 2023. Reasons: unreliable results or conclusions; concerns about the data; concerns about the peer review; concerns about the citations.

#### 3.2.3. Determine the Demand Point and Supply Point

It takes the streets and communities as the basic unit, the demand point is the demand location for education services, the neighborhood committee of each community is selected as the focus of the research, the supply point is the location that provides education services, and the secondary schools and primary schools in the old city of Ganzhou are selected. The latitude and longitude of the point and the supply point are obtained through the Zhanggong district government website and the python programming language by Baidu API interface.

The basic research unit of spatial autocorrelation analysis is community. The spatial distance between adjacent research units is small, which improves the scientificity of statistical analysis results. Accessibility analysis can not only obtain the proximity between supply point and demand point from space distance but also from time distance.

## 4. Results and Analysis

### 4.1. Accessibility from Community to Primary School

#### 4.1.1. Walking Accessibility

According to the building design specification for primary and secondary schools, the service range of primary schools should not be greater than 500 meters, but according to the 500-meter cost search radius, the distance from the school to most communities is greater than 500 meters, indicating that the coverage of the primary school in old districts is insufficient, hence expanding the search area range and taking the distance cost of 1000 meters as the search radius of schools and communities. On the whole, the accessibility of primary schools in the old district is divided significantly, and few people can enjoy the ideal state of accessibility. The communities with the highest accessibility are mainly Nanjing Road community, Shangshu Lane community, Datangbei, etc. The areas with the lowest accessibility are Land-temple community, Mulanjing community, Yaofuli community, Binjiang community, Yangmeidu community, and Yingjiao Shang communities, which have not found schools within 1000 meters and have extremely low accessibility. From the perspective of the streets in Table 1, Jiefang Street and Ganjiang Street have higher accessibility, while Nanwai Street and Dongwai Street have lower accessibility (Figure 4).

The adjacent relationship of spatial objects is the spatial relationship of basic phenomena. The introduction of the concept about spatial weight matrix into spatial statistical analysis is one of the important differences between spatial statistical analysis and traditional statistical analysis. When the Moran index I is greater than zero, it means that areas with similar eigenvalues have high or low-value clusters; when the Moran index I is less than zero, it means that areas with dissimilar eigenvalues have high or low-value or low high-value clusters. It can be seen from Figure 4 that according to the spatial autocorrelation analysis, the high-value gathering area is the junction of Ganjiang Street and Jiefang Street, and the low-value areas are mainly the southwest part of Nanwai Street and the northwest part of Dongwai Street (Figure 5).

The article "The Accessibility of Educational Public Service Facilities with Two-Step Mobile Search Taking Hetao District of Ganzhou City as an Example" was retracted in 2023. Reasons: unreliable results or conclusions; concerns about the data; concerns about the peer review; concerns about the citations.

#### 4.1.2. 5-Minute Driving Accessibility

Combined with the travel survey, the main travel options for primary schools are walking and driving by parents. Through route planning API with the Baidu map, two searches between primary school and community can be obtained within 5 minutes by driving to get the results. Compared with the cost by foot, the time cost of 5 minutes driving not only considers the road problem but also considers the traffic light situation and road congestion, which can more accurately reflect the real situation. On the whole, the high-value areas of primary school accessibility in old district are scattered, and the low-value areas are mainly distributed around the South Gate. The highest value areas mainly include Heping Road community, Jiankang Road community, Sankang Temple community, and Xiahaotang community, and the lowest value areas mainly include Land-Temple community, Xiaoyi Lane community, Renmin Lane community, Damiaoqian community, Taozi Garden communities, Nanwai community, Yingjiao Shang community, and Guandaoping community which indicate that the time cost of driving to primary school in these communities is relatively high. Judging from Table 2, the choice of driving shows that the accessibility of Jiefang Street is still the highest, and the accessibility of Ganjiang Street is relatively lower than that of walking, while the accessibility of Nanwai Street is relatively increased. It is relatively smooth and takes less time than Hongqi Avenue, while Ganjiang Street is more congested than Wenqing Road and other roads and takes more time by foot (Figure 6).

In Figure 7, with spatial autocorrelation analysis, due to the congestion of Wenqing Road and Nanhe Bridge, traffic accessibility in nearby areas is reduced, and low-value areas appear; high-value areas are distributed on Heping Road, Jiankang Road, Dagonglu, and Nanshijie community because of gathering around Houde Road Primary School and Dagonglu No.1 Primary School and so on nearby.

### 4.2. The Accessibility from Community to Secondary School

#### 4.2.1. Walk Accessibility of 1000-Meter to Secondary School

Combined with the travel survey, the travel mode of secondary school students is by foot and cycling. Cycling is the same as walking, without considering road and traffic congestion. Therefore, the walking mode is adopted as a research method. According to the building design specification of primary and secondary schools, the service range of secondary schools should not be greater than 1000 meters, so the distance cost of 1000 meters is conducted two times searching between the community and secondary school. On the whole, the high-value accessibility areas of old district are mainly centered in the core area, and the accessibility decreases from inside to outside of the city. The regional differentiation is obvious. There are not many people who can enjoy the ideal state of accessibility outside the city. Among them, the communities with the highest value mainly include Damiaoqian community, Diaoyutai Community and Yaofuli community. The lowest value areas are mostly in the northern and southeastern communities. Among them, there are many low-value areas, indicating that within the search threshold of 1000 meters, no schools are found in the low-value areas. From Table 3 by streets, the accessibility of Ganjiang Street is significantly higher than that of other streets, followed by Nanwai Street, Jiefang Street, and Dongwai Street which have lower accessibility (Figure 8).

The article "The Accessibility of Educational Public Service Facilities with Two-Step Mobile Search Taking Hetao District of Ganzhou City as an Example" was retracted in 2023. Reasons: unreliable results or conclusions; concerns about the data; concerns about the peer review; concerns about the citations.

From the spatial autocorrelation analysis, it can be more clearly seen that the Wenqing Road area at Nanmenkou has high spatial accessibility and high-high clusters, while low-low clusters appear in the north and south, reflecting the law of decreasing accessibility from the center to the surroundings (Figure 9).

#### 4.2.2. Walking Accessibility of 1500-Meter to the Secondary School

The search radius is expanded to 1500 meters, and the coverage area is further expanded, which can better reflect the distribution of accessibility planning. On the whole, the high-value accessibility areas in old district similar to 1000-meter search radius are mainly concentrated in the center of gravity, and the accessibility decreases from inside to outside of the city, but the extremely low value of accessibility decreases while the high-value areas are not. The continuous increase indicates that there are more communities and schools within the range of 1000 meters to 1500 meters. The high-value areas mainly include Hongcheng Alley, Xiaoyi Alley, Renmin Alley, Damiaoqian, Diaoyutai, Yaofuli, Dagonglu, Houde Road community, and low-value areas include Jianguo Road community, Nanwai community, Yingjiaoshang community, Laijiawei community. From Table 4, it can be seen that the accessibility of Ganjiang Street and Nanwai Street is relatively high, while the accessibility of Ganjiang and Dongwai Street is relatively low because of uneven education resources that No. 1, No. 3, No. 4, No. 7, and Affiliated Secondary School of Gannan Normal university are all concentrated in this area (Figure 10).

The article "The Accessibility of Educational Public Service Facilities with Two-Step Mobile Search Taking Hetao District of Ganzhou City as an Example" was retracted in 2023. Reasons: unreliable results or conclusions; concerns about the data; concerns about the peer review; concerns about the citations.

From the spatial autocorrelation analysis, it can be seen that due to the expansion of the search range, it can better reflect the real situation. The high-value area in the center has further increased, and the low-value area in the south has also increased, and the difference in accessibility between regions has increased. The decreasing law of the accessibility center to the surroundings is more obvious (Figure 11).

## 5. Conclusion and Discussion

### 5.1. Conclusion

The accessibility measurement to the spatial layout of educational service facilities of primary and secondary schools in the old city shows as follows:

1. The overall accessibility of primary and secondary schools in Ganzhou City is low. Most areas do not have sufficient and good education resources. At the same time, most residents fail to enjoy the equipment standards recommended by the Ministry of Education. The accessibility of primary school is expressed in geographical space as the high-value gathering area is the junction of Ganjiang Street and Jiefang Street, and the low-value areas are mainly in the southwest part of Nanwai Street and the northwest area of Dongwai Street, showing a scattered state. The accessibility of the secondary school shows decreasing accessibility from the center of the old city to the surroundings. The accessibility of the center is significantly higher than that of the north and south sides. The spatial distribution of accessibility is extremely uneven. It is liberated from the accessibility of the primary school at the street level; from the perspective of secondary school, Ganjiang Street has significantly higher accessibility than other streets, while Dongwai Street is significantly lower than other streets, indicating education resources in Hetao district of Ganzhou. There is a prominent contradiction between supply and demand
2. Compared with traditional methods, the spatial accessibility evaluation method of educational service facilities with the two-step mobile search of Internet map time cost and distance cost can evaluate the population of different travel modes based on the real-time traffic information of the city. By setting different time and distance impedances for secondary schools and primary schools in the old city of Ganzhou City, the spatial distribution of accessibility in Ganzhou's community under different travel modes is basically consistent with the public's spatial cognition, indicating the improved two-step approach introduced in this article. The mobile search method has certain application potential for the evaluation of the spatial accessibility of educational service facilities [1,15,16,24]

The article "The Accessibility of Educational Public Service Facilities with Two-Step Mobile Search Taking Hetao District of Ganzhou City as an Example" was retracted in 2023. Reasons: unreliable results or conclusions; concerns about the data; concerns about the peer review; concerns about the citations.

### 5.2. Suggestions

1. Follow the time and adapt measures to local conditions, rectify by divisions according to the general planning, and reserve land for short-term construction and long-term education in combination with the dynamic changes of urban population size and population structure. In view of the differentiation of the accessibility of secondary schools in the center and the periphery of the city, the city master planning should be used as a guide to appropriately control the expansion of schools in the central area and appropriately guide the relocation of some excessively concentrated schools to the surrounding areas. For the surrounding areas, an appropriate number of schools should be deployed in the future in order to meet the ever-expanding demand for schooling in the future, and the school should implement supporting educational facilities in the newly built community to ensure sufficient supply of degrees
2. Reasonably tap potential resources, scientifically make financial investment in educational facilities, and achieve a balance between the number and quality of future schools. Encourage existing teaching resources to rationally select locations in new urban areas and fringe areas and establish branch campuses. In view of the gap in accessibility between streets, the district government should strengthen research and implementation of the reasons to achieve balanced development of all streets.
3. Strengthen policy formulation and legislative guarantees to prevent the unbalanced spatial distribution of education resources from the root cause. Clarify the government's main role in the construction and management of educational service facilities, and clarify the responsibilities of various administrative departments in the construction of educational service facilities.

### 5.3. Outlook

This article combines Internet map data, two-step mobile search with spatial autocorrelation of ArcGIS. It not only pays attention to the interaction of urban public service facilities from supply but also calculates the potential services obtained by residents from demand, and it is a very effective tool to analyze the urban spatial structure and to obtain the fairness of the layout of public service facilities, but if it can be combined with the current school district policy, the evaluation unit is further refined to the residential area or the evaluation is based on the grid, and it will accurately evaluate the accessibility of educational service facilities in Hetao District of Ganzhou.

The article "The Accessibility of Educational Public Service Facilities with Two-Step Mobile Search Taking Hetao District of Ganzhou City as an Example" was retracted in 2023. Reasons: unreliable results or conclusions; concerns about the data; concerns about the peer review; concerns about the citations.

## Figures and Tables

**Figure 1:** Location of Ganzhou City.

**Figure 2:** Location of primary and secondary schools in Hetao district of Ganzhou city.

**Figure 3:** Baidu map data capture program example.

**Figure 4:** The spatial distribution of 1000-meter walk accessibility to primary school.

**Figure 5:** The spatial autocorrelation analysis of 1000-meter walk accessibility to primary school.

**Figure 6:** Spatial distribution of accessibility to primary schools for 5 minutes driving.

**Figure 7:** Spatial autocorrelation analysis of 5-minute reachability to primary school.

**Figure 8:** The spatial distribution of 1000-meter walk accessibility to secondary school.

**Figure 9:** The spatial autocorrelation analysis of 1000-meter walk to the secondary school.

**Figure 10:** Spatial distribution of 1500-meter walk accessibility to the secondary school.

**Figure 11:** Spatial autocorrelation of 1500-meter walk accessibility to the secondary school.

**Table 1:** Primary school accessibility of 1,000 meters by foot.

Street	Ganjiang	Jiefang	Dongwai	Nanwai
Accessibility	1.32	1.40	0.99	1.14

**Table 2:** Street accessibility to primary school for 5 minutes driving.

Street	Ganjiang	Jiefang	Dongwai	Nanwai
Accessibility	0.74	0.96	0.51	0.67

**Table 3:** The street accessibility of 1000-meters walk to the secondary school.

Street	Ganjiang	Jiefang	Dongwai	Nanwai
Accessibility	1.61	0.50	0.33	1.06

**Table 4:** Street accessibility of 1,500-meter walk to the secondary school.

Street	Ganjiang street	Jiefang street	Jiefang street	Jiefang street
Accessibility	1.37	0.85	0.36	1.04

## Data Availability

No data were used to support this study.

## References

[1] Deng L., Shao J. A., Guo Y. *Spatial accessibility of medical services in mountainous*.

[2] Wang H. F. (2011). *Quantitative Methods and Applications Based on GIS [M]*.

[3] Dai D. J. (2010). Black residential segregation, disparities in spatial access to health care facilities, and late-stage breast cancer diagnosis in metropolitan Detroit. *Health & Place*.

[4] Dai D. J. (2011). Racial/ethnic and socioeconomic disparities in urban green space accessibility: where to intervene?. *Landscape and Urban Planning*.

[5] Schuurman N., Bérubé M., Crooks V. A. (2010). Measuring potential spatial access to primary health care physicians using a modified gravity model. *Canadian Geographer/Le Géographe Canadien*.

[6] McGrail M. R., Humphreys J. S. (2009b). The index of rural access: an innovative integrated approach for measuring primary care access. *BMC Health Services Research*.

The article "The Accessibility of Educational Public Service Facilities with Two-Step Mobile Search Taking Hetao District of Ganzhou City as an Example" was retracted in 2023. Reasons: unreliable results or conclusions; concerns about the data; concerns about the peer review; concerns about the citations.

[7] Lu D. D. (1995). *Regional Development and its Spatial Structure [M]*.

[8] Wang Y. F., Zhang C. (2005). GIS and gravity polygon based service area analysis of public facility: case study of hospitals in Pudong New Area. *Economic Geography*.

[9] Chen L. X., Chen Z. (2008). Study on Therationality of Warm Guangzhou City Primary School Layout - Taking Hai Zhu District as an Example. *geographic China 2008 academic annual meeting*.

[10] Xiao Z. F. (2011). *Studies on Differentiation of Facility Space Secondary School in Xi’an City[D]*.

[11] Liu Z., Guo S. Q., Jin H. H. (2007). The two-step search method in mobile search GIS Beijing medical evaluation of spatial accessibility in application of. *J. the science of Surveying and mapping*.

[12] Deng L., Shao J. A., Guo Y. (2015). Spatial accessibility of medical services in mountainous regions based on modified two-step floating catchment area method: a case study of Shizhu County. *Chongqing. Progress in Geography*.

[13] Che L. H. (2013). Review on the measures and application of spatial accessibility to health care. *The Chinese Health Service Management*.

[14] Luo W., Wang F. (2003). Measures of spatial accessibility to health care in a GIS environment: synthesis and a case study in the chicago region. *Environment and Planning B: Planning and Design*.

[15] Luo W., Qi Y. (2009). An enhanced two-step floating catchment area (E2SFCA) method for measuring spatial accessibility to primary care physicians. *Health & Place*.

[16] MaGrail M. R., Humphreys J. S. (2009). Measuring spatial accessibility to primary care in rural areas: improving the effectiveness of the twostep floating catchment area method[J]. *Applied Geography*.

[17] Luo W., Whippo T. (2012). Variable catchment sizes for the two-step floating catchment area (2SFCA) method. *Health & Place*.

[18] Cheng Y., Liu M., Li M. Y. (2011). Spatial accessibility analysis of green space in suburb parks based on 2SFCA. *Central South Forest Inventory and Planning*.

[19] Hu R. S., Dong S. C., Hu H. (2012). A two-step floating catchment area (2SFCA) method for measuring spatial accessibility to primary healthcare service in China: a case study of Donghai County in Jiangsu Province[J]. *Progress in Geography*.

[20] Tao Z. L., Cheng Y. (2016). Research progress of the two-step floating catchment area method and extensions. *Progress in Geography*.

[21] Tao Z. L., Cheng Y., Dai T. Q. (2014). Measuring spatial accessibility to residential care facilities in Beijing. *Progress in Geography*.

[22] Wei Y., Xiu C. L., Gao R. (2014). Evaluation of green space accessibility of Shenyang using Gaussian based 2-step floating catchment area method. *Progress in Geography*.

The article "The Accessibility of Educational Public Service Facilities with Two-Step Mobile Search Taking Hetao District of Ganzhou City as an Example" was retracted in 2023. Reasons: unreliable results or conclusions; concerns about the data; concerns about the peer review; concerns about the citations.

[23] Zhang P. F., Cai Z. L., Zhang C. (2015). Potential spatial accessibility to urban scenic spots based on E2SF- CA. *Journal of Geomatics*.

[24] Wang J. F., Zhang T. L., Fu B. J. (2016). A measure of spatial stratified heterogeneity. *Ecological Indicators*.

